The article "Pain Management of Hallux Valgus Surgery Is Achieved by Cocktail Therapy" was published in 2022. Journal: Evid Based Complement Alternat Med.

# Pain Management of Hallux Valgus Surgery Is Achieved by Cocktail Therapy

**DOI:** 10.1155/2022/1084815

**Published:** 2022-09-02

**Authors:** Jiewei Xie, Junlang Zhu, Yiyin Xu, Mengli Chen, Haiyun Chen, Kaiping Yuan, Dingkun Lin

**Affiliations:** ^1^Department of Trauma and Foot-Ankle Surgery, Guangdong Provincial Hospital of Chinese Medicine, Guangzhou 510120, China; ^2^Department of Trauma and Foot-Ankle Surgery, The Second Affiliated Hospital of Guangzhou University of Chinese Medicine, Guangzhou 510120, China; ^3^Department of No. 3 Orthopaedics, Dongguan City Houjie Hospital, Dongguan 523962, China

## Abstract

**Background:**

Hallux valgus is a relatively common forefoot disease in clinical practice. The aim of our study was to assess the role of local cocktail drugs and postoperative pain after hallux valgus surgery.

**Methods:**

A retrospective case-control study was conducted to analyze 75 moderate to severe hallux valgus patients from June 1, 2018 to December 1, 2019. All patients were divided into cocktail and control groups according to whether the cocktail therapy was used or not after the operation. The anesthesiologist did not provide analgesic treatment other than nerve block anesthesia and intravenous anesthesia, such as analgesic pumps. The operative region of the cocktail group received a mixture of 10 ml of 0.75% ropivacaine, 10 ml of flurbiprofen axetil injection, and 1 ml of compound betamethasone injection, whereas the control group received nothing in the surgical spot. We recorded patients' VAS scores preoperatively and at 6, 24 hours postoperatively; the length of hospital stay and the number of hospitalization expenses; the scores of Kolcaba comfort level; and the scores of Pittsburgh sleep quality.

**Result:**

There was no significant difference in age or sex between the two groups. The VAS scores at 6 and 24 hours postoperatively were significantly lower in the cocktail group. The average length of hospital stay was 8.24 days in the control group and 3.73 days in the cocktail group. The average total hospitalization cost of the control group was ¥28285.16, and that of the cocktail group was ¥22366.31. In expenses of total hospitalization costs, the cocktail group was lower than the control group. Kolcaba's comfort various scores and the total score of the cocktail group were higher than the control group. The total score of PSQI and all dimensions in the experimental group were lower than those in the control group.

**Conclusion:**

We found a significant difference in the results of postoperative pain management except for age, sex, and hospitalization expenses. After hallux valgus surgery, inject cocktail drugs around the first metatarsophalangeal joint did reduce postoperative pain level. *Level of Evidence*. Level III, case-control study.

The article "Pain Management of Hallux Valgus Surgery Is Achieved by Cocktail Therapy" was published in 2022. Journal: Evid Based Complement Alternat Med.

## 1. Introduction

Hallux valgus (HV) is a progressive foot deformity presenting with lateral deviation of the hallux and medial deviation of the first metatarsal head [1]. HV is very common, affecting approximately 23% of adults [2]. To achieve the normal function of the foot, it is necessary to achieve normal three-point plantar weight bearing. Furthermore, HV is a common forefoot abnormality with a prevalence of up to 23% in the general population [3]. Patients with HV have altered stress on the toe and increased postural sway while walking, and their general foot function and participation in physical activities are adversely affected.

Foot and ankle surgeons have been seeking a minimally invasive, safe, effective, and reliable treatment for HV [4]. The minimally invasive operation of HV can reduce the degree of postoperative pain. In recent years, some foot and ankle surgeons have used a new invasive intramedullary nail device to treat mild to severe hallux valgus, achieving good treatment effects and low postoperative complications and recurrence rates [5, 6]. Chen et al. followed up on 308 patients who had undergone HV surgery and found that 31% still had residual pain six months after surgery [7]. HV correction is painful and inconvenient. Pain relief is the primary goal of HV surgery, malformation correction is the secondary goal [8]. The analgesic regimen for HV orthopedics should include, in the absence of contraindication, paracetamol and a nonsteroidal anti-inflammatory drug or cyclo-oxygenase-2 selective inhibitor administered preoperatively or intraoperatively and continued postoperatively, along with systemic steroids and postoperative opioids for rescue analgesia [6]. Patients with HV experience moderate to severe pain for 2-3 days after surgery [9]. Acute pain after HV surgery is a physiological and psychological reaction to the tissue damage caused by the operation. If the pain control after HV surgery is poor, it can lead to respiratory and cardiovascular complications, which is not conducive to the postoperative recovery of patients, resulting in increased hospital stay and cost. Local corticosteroid injections, which can significantly promote functional recovery and pain relief due to their fast-acting anti-inflammatory effects, reduce local swelling. Local anesthetic use for wound infusions, single injections, and continuous nerve blocks for postoperative analgesia is well established [10]. Surgical general anesthesia-assisted local infiltration anesthesia is increasingly being used as an adjunct to perioperative pain management to reduce the amount of analgesic required after surgery [11, 12]. Effective analgesic methods, postoperative patients can use less opioid doses while also reducing common side effects such as respiratory depression, sedation, nausea, constipation, itching, and urinary retention. The cocktail therapy proposed in this study is injected by the surgeon under direct vision with a small dosage and had no adverse reactions so far. It can reach the painful site and eliminate the pain from the source. The optimal forms of analgesia are effective, simple to administer, acceptable to the patient, and have minimal side effects. Compared with ankle nerve block [13], it is easier to promote learning without increasing the risk of infection. The aim of our study was to assess the role of local cocktail drugs and postoperative pain after hallux valgus surgery.

The article "Pain Management of Hallux Valgus Surgery Is Achieved by Cocktail Therapy" was published in 2022. Journal: Evid Based Complement Alternat Med.

## 2. Materials and Methods

This study is a retrospective controlled study. We conducted an analysis of 75 hallux valgus patients and performed osteotomy combined with lateral soft tissue release of the foot from June 1, 2018 to December 1, 2019. All patients were divided into a treatment group (41 patients) and control group (34 patients) according to whether cocktail therapy was used or not after the operation. All patients had a one-sided operation.

### 2.1. Inclusion Criteria

The inclusion criteria were as follows: aged 18–85 years, American Society of Anaesthesiologists (ASA) score of I-II, no peripheral neuropathy or allergy to local anesthetics and cortisol, and no history of foot procedure measured by preoperative weight-bearing radiographs of the affected foot, moderate HV: 20° < Hallux valgus angle (HVA) ≤ 40°, 13° < inter metatarsal angle (IMA) ≤ 16°; Severe HV: HVA > 40°, IMA > 16°, the presence of the first metatarsophalangeal joint medial pain, or combined with the second, third metatarsophalangeal pain with callose patients, after conservative treatment ineffective; and radiographs show poor articulation or dislocation of the metatarsophalangeal joint.

### 2.2. Exclusion Criteria

The exclusion criteria were as follows: severe degenerative arthritis of the first metatarsophalangeal joint; patients with severe osteoporosis; local skin ulcer infection; and HV caused by rheumatoid arthritis, flat feet, trauma, neuromuscular disease. Furthermore, we also excluded patients with peripheral circulatory disorders, diabetes, and rheumatoid diseases; skin lesions of the foot; allergy to local anesthetic; and patients using analgesics 10 days prior to surgery.

The cocktail group received a mixture of 10 ml of 0.75% ropivacaine, 10 ml of flurbiprofen axetil injection, 1 ml of compound betamethasone injection, and a total of 21 ml, whereas the control group received no drugs in the surgical spot. We did not use betamethasone in patients with a history of diabetes. We defined the term “cocktail” in this study as a mixture of a local anesthetic, flurbiprofen, and corticosteroid. In both the treatment group and the control group, from the day after HV surgery, pain management was performed by administering nonsteroidal anti-inflammatory drugs at 180 mg/d for 7 days and tramadol hydrochloride at 2 mg/kg for moderate to severe pain. All patients undergoing HV surgery were assessed by the nurse with the Visual Analogue Score (VSA), Kolcaba Comfort Score, and Pittsburgh Sleep Quality Index Score (PSQI). We evaluated patients' visual analog scale (VAS) scores preoperatively and at 6 and 24 hours postoperatively and the Pittsburgh sleep scores, postoperatively.

The article "Pain Management of Hallux Valgus Surgery Is Achieved by Cocktail Therapy" was published in 2022. Journal: Evid Based Complement Alternat Med.

## 3. Evaluated Parameters

We evaluated patients' VAS scores preoperatively and at 6 and 24 hours postoperatively. Finally, we evaluated the length of hospital stay and the number of hospitalization expenses; the scores of the Kolcaba comfort level; and the scores of Pittsburgh sleep quality. We compared these items retrospectively between the two groups.

## 4. Surgical Procedures

After successful anesthesia, patients were placed in a supine position with a tourniquet at the root of the thigh. A 1 cm incision was made on the lateral side of the first metatarsophalangeal joint, and the sapoid suspensory ligament and adduction tendon of the great toe were cut. The joint capsule was released appropriately so that the passive adduction of the great toe was at least 25°. A partial metatarsal incision was made on the medial side of the great toe. The joint capsule was opened in a shuttle shape to expose the osteophyte and metatarsal bone, and the osteophyte was removed. The osteotomy vertex was established at 0.8–1 cm and 1/3 above the articular surface of the head, and the direction of the fourth metatarsal bone was used as the osteotomy direction. Mini-swing saw “*V*” shaped 70°∼80° angle osteotomy, forming a short upper arm, long lower arm improved osteotomy [14]. We clamp the diaphysis of the first metatarsal bone with a tissue forceps, traction the thumb, and push the distal bone 5–8 mm laterally to the proper position of orthosis, and clamp the distal part of the lower arm with vascular forceps to prevent the elevation of the metatarsal bone. Two Kirschner wires with a diameter of 1 mm were used for temporary fixation, and cloth forceps were used for temporary fixation of the medial joint capsule without tension. The second fluoroscopic observation confirmed that the orthopedic position was appropriate and screwed in one-two 3.0 full-thread headless compression screws for fixation, and the inner convex part was smoothened with a swing saw [15, 16]. If a poor metatarsal-toe joint is found, or a DMMA angle ≥9° is found (as assessed by preoperative measurements and surgical appearance and fluoroscopy), a closed wedge osteotomy (Akin osteotomy) is performed on the base medial side of the proximal phalangeal of the first big toe. For patients with preoperative hypermobility in the first tarsometatarsal joint, a Lapidus procedure involving arthrodesis of the joint was performed [17, 18]. The modified McBride soft tissue procedure was also performed in all patients, a 2 cm incision was made on the lateral side of the first metatarsophalangeal joint, and the sesamoid suspensory ligament and adductor tendon of the first toe were severed, appropriately releasing the joint capsule to allow passive adduction of the first toe less than 25°. The cocktail of drugs was injected into the periosteum, joint capsule, and subcutaneously (Figure 1). The incision was rinsed, the HV was about 3°, and the medial joint capsule and incision were sutured with 3-0 absorbable sutures without tension. Sutured fascia, subcutaneous, sterile gauze bandaging, keeping the hallex straight and fixed, with moderate tension inward, to prevent the compressed joint capsule from splitting.

The article "Pain Management of Hallux Valgus Surgery Is Achieved by Cocktail Therapy" was published in 2022. Journal: Evid Based Complement Alternat Med.

## 5. Statistical Analysis

*T* test was used for quantitative data conforming to the normal distribution, and the rank sum test was used for data not conforming to normal distribution. *P* < 0.05 was considered statistically significant to compare differences in outcomes between the two groups. SPSS Statistics for Windows (version 22.0; IBM, Armonk, NY, USA) was used for all statistical analyses, and the results are presented as mean values. If normality of continuous variables was not assumed, nonparametric analysis including the Mann–Whitney *U* test and Wilcoxon signed-rank test was used instead. The Chi-square test and Fisher exact test (if any expected value lower than 5 was observed) were used for categorical data.

## 6. Results

All patients were divided into a treatment group (41 patients) and a control group (34 patients) according to whether cocktail therapy was used or not after the operation. All patients had a one-sided operation. Nobody experienced infection and delayed wound healing as adverse effects in the two groups. There was no significant difference in general clinical information between the two groups (*P* > 0.05). As shown in Table 1, the average length of hospitalization was 8.24 days in the control group and 3.73 days in the cocktail group, and the difference was statistically significant (*P* < 0.05). The average total hospitalization cost of the control group was ¥28285.16 and that of the cocktail group was ¥22366.31 (*P* > 0.05). The average total hospitalization cost of the cocktail group was lower than that of the control group, and the difference was statistically significant (*P* < 0.05) (Table 1). The VAS score of the cocktail group was lower than that of the control group at 6 hours and 24 hours after surgery, the difference was statistically significant (*P* < 0.05) (Table 2). The Kolcaba comfort scores and total scores in the cocktail group were higher than those in the control group, with a statistical significance (*P* < 0.05) (Table 3). The PSQI total score and all dimension scores of the cocktail group were lower than those of the control group, with a statistical significance (except daytime function) (*P* < 0.05) (Table 4).

The article "Pain Management of Hallux Valgus Surgery Is Achieved by Cocktail Therapy" was published in 2022. Journal: Evid Based Complement Alternat Med.

## 7. Discussion

In recent years, local injection of incision analgesia has attracted the attention of orthopedic surgeons [19]. This study investigated painless technology in HV corrective surgery. We provide a convenient and effective pain management technique for foot and ankle surgeons. The technique of ankle nerve block requires the surgeon to be familiar with the anatomy of the foot and ankle nerves. Ankle nerve blocks are relatively complicated, and some patients may experience transient nerve palsy [13]. Good postoperative analgesic effects can not only reduce postoperative stress response and reduce cardiovascular load but also provide good conditions for postoperative rehabilitation and joint function recovery [20]. Although minimally invasive and improved surgical methods are mostly used in HV surgery now, postoperative pain management is of vital significance for early recovery [6]. A femoral-sciatic nerve block or ankle block regional anesthesia was safe and effective in reducing postoperative pain, with a low incidence of chronic pain syndrome. However, it is just for mild-to-moderate HV (without concomitant forefoot procedures: e.g., hammertoe correction, claw toe correction) [21]. A bigger drawback is that the surgeon cannot use a tourniquet for this type of analgesia. There are two orthopedic surgeons in our hospital with similar seniority, who have accumulated rich experience in HV orthopedic surgery. One orthopedic surgeon administered a cocktail of analgesics to the area after surgery, while the other never used cocktails. Despite this, the two doctors have the same principles, concepts, and methods of surgical treatment for HV. There are two main reasons for pain after HV surgery: (1) pain generated by surgical incision: this kind of pain is received by skin nociceptors and transmitted to the cerebral cortex through spinal cord posterior horn cells, which is a superficial sensation and most patients describe it as acute pain. (2) Pain from the foot: the operation around the forefoot and middle foot leads to bleeding around the operative mouth of the foot, blood accumulation, tissue edema, and other stimuli to the proprioceptors, which are passed into the thalamus through the thin and wedge bundles, belonging to the deep feeling, and the patient describes it swelling pain. Therefore, the incision pain management for patients with HV surgery should start from the above two aspects, not only to solve the acute pain in the wound but also to solve the swelling pain caused by blood accumulation and tissue swelling in the soft tissue.

The article "Pain Management of Hallux Valgus Surgery Is Achieved by Cocktail Therapy" was published in 2022. Journal: Evid Based Complement Alternat Med.

Flurbiprofen is a class of nonsteroidal anti-inflammatory drugs of propionic acid, which is one of the powerful antipyretic and analgesic drugs. Its use in advanced analgesia can effectively relieve postoperative pain and it has a good anti-inflammatory effect. Ropivacaine is a new long-acting local anesthetic, which blocks nerve excitation conduction by inhibiting sodium ion channels [22, 23]. Compound betamethasone is a glucocorticoid drug, which can significantly reduce the serum C-reactive protein content and white blood cell number and can play a synergistic analgesic and anti-inflammatory effect when used in combination with flurbiprofen [23]. For diabetic patients, the safety concerns of using glucocorticoids mainly lie in incision infection and postoperative hyperglycemia. Good postoperative analgesia is helpful to stabilize postoperative blood glucose fluctuations and counteract the elevated blood glucose effect of glucocorticoids, so there is no significant increase in perioperative blood glucose levels in patients using glucocorticoids [24]. A low concentration of ropivacaine has a blocking effect on sensory-motor separation, and patients can get off the ground earlier, which can effectively cooperate with rehabilitation training. Given the adverse reactions associated with opioids, such as postoperative nausea and vomiting, as well as studies of the harms of current opioids, opioids should be considered as rescue analgesics only if nonsteroidal anti-inflammatory drugs fail to provide adequate pain relief [25, 26]. The cocktail formula used in general joint surgery contains epinephrine. It is generally believed that epinephrine should be avoided when local anesthesia is implemented in the peripheral blood-carrying organs such as fingers, toes, ears, and nose, in order to prevent tissue ischemia and necrosis caused by constriction of peripheral blood vessels [27].

The article "Pain Management of Hallux Valgus Surgery Is Achieved by Cocktail Therapy" was published in 2022. Journal: Evid Based Complement Alternat Med.

We defined the best cocktail analgesic drugs in this study as a mixture of a local anesthetic, flurbiprofen, and corticosteroid. On the basis of conventional anesthesia, we injected a “cocktail” around the surgical area after HV surgery and found that in the cocktail group, the VAS score of foot pain was significantly reduced, and the amount of time and money spent in the hospital was less, the total score of PSQI in all dimensions was lower, and the Kolcaba comfort score was higher. In addition, the retrospective controlled study of Qeng et al. in the field of foot and ankle surgery also had fewer patients in the control group than in the treatment group [28]. Because this study is a retrospective controlled study in the field of foot and ankle surgery, it is impossible to control the same number of people in the control group and the treatment group.

There are some limitations to this study. First, this was a retrospective study with a small sample size due to patients being excluded to eliminate the impact of other foot deformities on the clinical efficacy and with a short follow-up time. In addition, this study also has the problems of a small sample size and short follow-up time. Besides, it is not clear if a nerve block during surgery before the surgery could reduce postoperative pain, too. In the future, a prospective clinical trial with a larger sample size should be conducted in the future to further validate the findings of this study.

## 8. Conclusion

We compared with or without cocktail therapy after hallux valgus surgery and found a significant difference in the results of postoperative pain management except for age, sex, and hospitalization expenses. The analgesic duration of cocktail analgesia was much longer than that of conventional surgical anesthesia. In summary, injecting cocktail drugs around the operation areas did reduce the postoperative pain level. Cocktail analgesia allows patients to be as comfortable as possible after HV surgery. The cocktail may be beneficial for HV surgery patients, though some limitations might weaken the validity of these findings. More RCTs of high quality and more carefully designed clinical trials are recommended to generate a high level of clinical evidence to confirm these findings.

## Figures and Tables

**Figure 1:** The cocktail drugs was injected from the periosteum (a), joint capsule (b), and subcutaneously (c).

**Table 1:** The average length of hospital stay and total hospitalization cost between two groups.

Group	Hospital stay (days)	Hospitalization cost (¥)
Control group (*n* = 34)	8.24 ± 2.797	28285.16 ± 15780.498
Cocktail group (*n* = 41)	3.73 ± 1.597^*∗*^	22366.31 ± 5008.494
*Z* value	−6.52	−9.90
*P* value	*P* ≤ 0.01	0.322

The article "Pain Management of Hallux Valgus Surgery Is Achieved by Cocktail Therapy" was published in 2022. Journal: Evid Based Complement Alternat Med.

**Table 2:** Pain intensity measured by VAS in the control and cocktail groups.

Group	VAS score (6 hours after surgery)	VAS score (24 hours after surgery)
Control group (*n* = 34)	4.56 ± 15.22	2.94 ± 1.391
Cocktail group (*n* = 41)	1.32 ± 0.471^*∗*^	0.9 ± 0.3^*∗*^
*Z* value	−7.042	−6.938
*P* value	*P* ≤ 0.01	*P* ≤ 0.01

**Table 3:** Comparison of the postoperative Kolcaba comfort level between the two groups.

Group	Physiology	Psychology	Spirit	Social culture	Total score
Control group (*n* = 34)	13.85 ± 1.417	30.12 ± 3.131	19.76 ± 2.641	18.76 ± 1.075	82.5 ± 7.102
Cocktail group (*n* = 41)	15.49 ± 2.146^*∗*^	32.05 ± 3.316^*∗*^	22.76 ± 1.374^*∗*^	19.56 ± 0.776^*∗*^	89.85 ± 5.773^*∗*^
*Z* value	−3.832	−2.331	−5.079	−2.898	−4.580
*P* value	*P* ≤ 0.01	*P* ≤ 0.01	*P* ≤ 0.01	*P* ≤ 0.01	*P* ≤ 0.01

**Table 4:** Comparison of postoperative sleep quality between the two groups.

Group	Time in bed	Sleep time	Sleep efficiency	Sleep quality	Sleep disorders	Use of sleeping pills	Daytime function	Total score
Control group (*n* = 34)	0.62 ± 0.697	1.5 ± 0.929	1.12 ± 0.729	1.41 ± 0.925	1.74 ± 0.828	0.88 ± 0.537	0.5 ± 0.663	7.76 ± 1.759
Cocktail group (*n* = 41)	0.22 ± 0.525^*∗*^	0.78 ± 0.69^*∗*^	0.59 ± 0.741^*∗*^	0.83 ± 0.803^*∗*^	1.07 ± 0.648^*∗*^	0.44 ± 0.594^*∗*^	0.29 ± 0.461	4.22 ± 2.77^*∗*^
*Z* value	−2.942	−3.351	−3.025	−2.664	−3.379	−3.33	−1.292	−5.207
*P* value	*P* ≤ 0.01	*P* ≤ 0.01	*P* ≤ 0.01	*P* ≤ 0.01	*P* ≤ 0.01	*P* ≤ 0.01	*P* ≤ 0.01	*P* ≤ 0.01

## Data Availability

The figures and table data used to support the findings of this study are available from the corresponding author upon request.
